# Endothelin-1 Inhibits Prolyl Hydroxylase Domain 2 to Activate Hypoxia-Inducible Factor-1α in Melanoma Cells

This article has been retracted.

**DOI:** 10.1371/journal.pone.0011241

**Published:** 2010-06-21

**Authors:** Francesca Spinella, Laura Rosanò, Martina Del Duca, Valeriana Di Castro, Maria Rita Nicotra, Pier Giorgio Natali, Anna Bagnato

**Affiliations:** 1 Laboratory of Molecular Pathology, Regina Elena National Cancer Institute, Rome, Italy; 2 Molecular Biology and Pathology Institute, National Research Council, Rome, Italy; Roswell Park Cancer Institute, United States of America

## Abstract

**Background:**

The endothelin B receptor (ET_B_R) promotes tumorigenesis and melanoma progression through activation by endothelin (ET)-1, thus representing a promising therapeutic target. The stability of hypoxia-inducible factor (HIF)-1α is essential for melanomagenesis and progression, and is controlled by site-specific hydroxylation carried out by HIF-prolyl hydroxylase domain (PHD) and subsequent proteosomal degradation.

**Principal Findings:**

Here we found that in melanoma cells ET-1, ET-2, and ET-3 through ET_B_R, enhance the expression and activity of HIF-1α and HIF-2α that in turn regulate the expression of vascular endothelial growth factor (VEGF) in response to ETs or hypoxia. Under normoxic conditions, ET-1 controls HIF-α stability by inhibiting its degradation, as determined by impaired degradation of a reporter gene containing the HIF-1α oxygen-dependent degradation domain encompassing the PHD-targeted prolines. In particular, ETs through ET_B_R markedly decrease PHD2 mRNA and protein levels and promoter activity. In addition, activation of phosphatidylinositol 3-kinase (PI3K)-dependent integrin linked kinase (ILK)-AKT-mammalian target of rapamycin (mTOR) pathway is required for ET_B_R-mediated PHD2 inhibition, HIF-1α, HIF-2α, and VEGF expression. At functional level, PHD2 knockdown does not further increase ETs-induced *in vitro* tube formation of endothelial cells and melanoma cell invasiveness, demonstrating that these processes are regulated in a PHD2-dependent manner. In human primary and metastatic melanoma tissues as well as in cell lines, that express high levels of HIF-1α, ET_B_R expression is associated with low PHD2 levels. In melanoma xenografts, ET_B_R blockade by ET_B_R antagonist results in a concomitant reduction of tumor growth, angiogenesis, HIF-1α, and HIF-2α expression, and an increase in PHD2 levels.

**Conclusions:**

In this study we identified the underlying mechanism by which ET-1, through the regulation of PHD2, controls HIF-1α stability and thereby regulates angiogenesis and melanoma cell invasion. These results further indicate that targeting ET_B_R may represent a potential therapeutic treatment of melanoma by impairing HIF-1α stability.

## Introduction

In melanoma hypoxic setting, the upregulation of hypoxia-inducible factor (HIF)-1α, the main transcriptional factor that allows cellular adaptation to hypoxia, is associated with vascular endothelial growth factor (VEGF) expression, neovascularization, poor prognosis, and resistance to therapy [1]–[4]. Moreover, it has been demonstrated that HIF-1α stabilization is essential for oncogene-driven melanocyte transformation and early stages of melanoma progression [5]. The HIF transcriptional activity is mediated by two distinct heterodimeric complexes composed by a constitutively expressed HIF-β subunit bound to either HIF-1α or HIF-2α [6]–[9]. HIF-α subunit is constantly transcribed and translated, but under normal oxygen conditions, undergoes hydroxylation at two prolyl residues located in the oxygen-dependent degradation domain (ODDD). The hydroxylation allows interaction of HIF-α with the E3-ubiquitin ligase, containing the von Hippen-Lindau protein (pVHL), and subsequently polyubiquitinated, leading to destruction by the proteasome [10], [11].

The increase of HIF-1α subunit is critically dependent on the three prolyl hydroxylase domain proteins termed PHD1, PHD2, and PHD3, that hydroxylate prolines Pro402 and Pro564 in the ODDD of HIF-1α [10]–[13]. Experimental evidences indicate that PHD2 is the major PHD isoform controlling HIF-1α protein stability [14]. In response to hypoxia, HIF-1 binds a conserved DNA consensus sequence known as the hypoxia-responsive element (HRE) on promoters of genes encoding molecules controlling tumor angiogenesis, such as *endothelin-1* (*ET-1*), *VEGF*, and *erythropoietin*, in different tumor cells [6], [15], [16].

Recent studies have demonstrated that endothelins (ETs) and endothelin B receptor (ET_B_R) pathway plays a relevant role in melanocyte transformation and melanoma progression [17], [19]. The ET family consists of three isopeptides, ET-1, ET-2, and ET-3, which bind to two distinct subtypes, ET_A_R and ET_B_R, of G protein-coupled receptors [20]. Gene expression profiling of human melanoma biopsies and cell lines indicated ET_B_R as a tumor progression marker associated with an aggressive phenotype [21], [22]. Activation of ET_B_R occurs since the early stages of melanoma progression allowing tumor cells to escape growth control, and to invade indicating that ET_B_R may represent a potential therapeutic target for melanoma [23]–[25]. Among emerging evidences underlining the contribution of ET-1 axis to tumor progression is the finding that ET-1 can influence the accumulation of HIF-1α in different cell types, including melanoma, ovarian and breast cancer and lymphatic endothelial cells [16], [25]–[28]. However the detailed molecular mechanism responsible for the HIF-1α increase remains unknown.

Here we demonstrate that in melanoma cells in normoxic conditions ET_B_R activation induces HIF-1α and HIF-2α accumulation, activity, and target gene expression by inhibiting HIF-α degradation. These effects are accompanied by inhibition of PHD2 protein levels and promoter activity, associated with increased angiogenic effects and melanoma cell invasion. Finally, we demonstrated that *in vivo* the inhibition of tumor growth and neovascularization by treatment with a selective ET_B_R antagonist is associated with an increase in PHD2 protein levels. Therefore, our findings identify the molecular mechanism by which ET-1 axis controls HIF-1α stabilization through the involvement of PHD2 degradation pathway, providing further support to the notion that ET_B_R blockade may offer a potential tool for melanoma treatment.

## Results

### ETs induce HIF-1α and HIF-2α accumulation and activity through ET_B_R

HIF-1α and HIF-2α have been proposed to function as key factors in angiogenesis and their expression has been associated with VEGF expression in human melanoma [4]. In this study we investigated the role of ET-1 axis on both HIF-1α and HIF-2α induction and transcriptional activity in melanoma cells. In primary (1007) and metastatic (SKMel28, M10, Mel120, M14) melanoma cell lines cultured in normoxic conditions ET-1 or ET-3 markedly increased HIF-2α protein levels, that paralleled HIF-1α accumulation, in all cell lines (Figure 1A). Moreover ET-2, similarly to ET-1 and ET-3, was able to induce HIF-1α and HIF-2α protein accumulation (Figure 1B). The inhibitory effect produced by two different ET_B_R pharmacological inhibitors, BQ788, a peptide antagonist, and A-192621, a nonpeptide ET_B_R antagonist, as well as by ET_B_R silencing by specific siRNA showed that ET_B_R is the relevant receptor that controls HIF-1α and HIF-2α protein accumulation (Figure 1B and Figure S1A). In melanoma cells, ET-1 induced a dose- and time-dependent induction of HIF-1α and HIF-2α reaching the maximum at 100 nM following 16–24 h stimulation (Figure S1B). Similarly, ET-3 stimulated a dose- and time-dependent HIF-1α accumulation, whereas an unrelated peptide not implicated in angiogenesis [29] was unable to induce it (Figure S1C). To determine whether ETs-induced HIF-1α is transcriptionally active, we transfected melanoma cells with a luciferase reporter gene driven by three specific HRE. ET-1 or ET-3 treatment resulted in a significant increase (p<0.005) in HIF-1α-induced luciferase reporter activity, that was blocked by BQ788, as well as by ET_B_R siRNA (Figure 1C). The ET-1-induced HIF-1α transcriptional activation was further investigated by analyzing the effect of ET-1 or ET-3 on VEGF. The increase in HIF-1α and HIF-2α protein levels in the presence of ET-1 or ET-3 or hypoxia paralleled those of VEGF (Figure 1D). When HIF-1α or HIF-2α were silenced by specific siRNA, ETs- or hypoxia-induced VEGF expression was inhibited (Figure 1D), indicating that either HIF-1α or HIF-2α can regulate target genes, such as VEGF, in melanoma cells.

**Figure 1:** ETs induce HIF-1α and HIF-2α accumulation and activation through ET_B_R. HIF-1α or HIF-2α protein expression was analysed in cell lysates from: **A**. Primary 1007, and metastatic, SKMel28, M10, Mel120, and M14 melanoma cells treated with ET-1 or ET-3; **B**. 1007 cells treated with ET-1, ET-2 or ET-3 or with BQ788 or A-192621, in combination with ET-1, or transfected with scRNA or ET_B_R siRNA and treated with ET-1 for 16 h. **C**. 1007 cells were transiently transfected with HRE-luciferase promoter construct in the presence of either ET-1 or ET-3 or in combination with BQ788, or transfected with ET_B_R siRNA for 16 h. Luciferase activity was measured and expressed as fold-increase, Bars, ± SD. *, p<0.005 compared to control; **, p<0.001 compared to ET-1 or ET-3. **D**. 1007 cells transfected with scRNA or with HIF-1α siRNA or HIF-2α siRNA were stimulated with either ET-1 or ET-3 or hypoxia (H) for 16 h, and cell lysates were analyzed for protein expression.

### ETs induce HIF-1α stability by impairing HIF-1α hydroxylation

To asses whether ET-1 axis stabilizes HIF-1α protein, we monitored the decay of HIF-1α after blockade of protein synthesis with cyclohexamide (CHX). Melanoma cells were stimulated for 24 h either with hypoxia, or with ET-1 and then treated with CHX under normoxic conditions for the indicated times. In these conditions the decay of HIF-1α protein was observed within 120 min and was completely undetectable by the end of 240 min (Figure 2A). When the cells were treated for 24 h with ET-1 and then with CHX and ET-1, the increased levels of HIF-1α remained constant up to 240 min, demonstrating that ET-1 is able to maintain stability of HIF-1α in normoxia by slowing down its degradation. The proteosome inhibitor MG132 protected the HIF-1α subunit from proteosome degradation and this effect was further increased in the presence of ET-1, indicating that ET-1, similarly to MG132, inhibits HIF-1α degradation (Figure 2B). Because hydroxylation at the 4-position of Pro402 and Pro564 within the ODDD of HIF-1α is responsible for its degradation under normoxia [10], we further investigated the role of ET-1 on the stability of HIF-1α by transfecting melanoma cells with a reporter plasmid expressing HIF-1α ODDD fused with luciferase (CMV-Luc-ODDD). Following the transfection, cells were stimulated for different times with ET-1 or cultured under hypoxia. As shown in Figure 2C, luciferase-ODDD stabilization increased in a time-dependent manner after stimulation with ET-1 or hypoxia, with maximal levels attained at 16h. Dose-response analysis showed that CMV-Luc-ODDD stability increased progressively reaching 3,5 fold induction compared to control at 100 nM ET-1 (Figure S2). ET-1 or ET-3-induced effect on HIF-1α stability was mediated by ET_B_R, as demonstrated by the inhibitory effect of BQ788 (Figure 2D). Altogether these results indicate that ET-1 axis increases HIF-1α protein stabilization by impairing HIF-1α hydroxylation.

**Figure 2:** ETs induce HIF-1α protein stability by impairing HIFα hydroxylation. **A**. 1007 cells were cultured under normoxic conditions (C) or exposed to hypoxia (H) or treated with ET-1 for 24 h. Following stimulation of CHX alone or in combination with ET-1 for the indicated times. **B**. 1007 cells were treated with MG132 alone or in combination with ET-1 for 24 h. **C**. 1007 and SKMel28 cells were transfected with CMV-Luc- ODDD construct and stimulated as indicated. Luciferase activity was expressed as fold induction. Bars, ± SD. *, p<0.004 compared to control. **D**. Cells transfected as in A were treated with ET-1 or ET-3 alone or in combination with BQ788 for 16 h. Bars, ± SD. *, p<0.005, compared to control; **, p<0.001 compared to ET-1 or ET-3.

### ETs inhibit PHD2 expression and promoter activity to stabilize HIF-α

To investigate the oxygen sensing mechanism that regulates HIF-1α stability, we evaluated the effect of ET-1 on PHD1, PHD2, and PHD3 protein levels in melanoma cells. While ET-1 produced minor changes on PHD1 and PHD3 expression, this peptide significantly decreased PHD2 protein levels in a time-dependent manner, and this effect was abolished by the presence of BQ788 (Figure 3A,B). Next to assesses how ET_B_R, HIF-1α, HIF-2α and PHD2 protein expression relate to one another, we examined their expression in five melanoma cell lines in the presence of ET-1. Primary and metastatic melanoma cells with high ET_B_R activation, following stimulation with ET-1, showed increased HIF-1α and HIF-2α protein associated with decreased PHD2 levels thus indicating that activation of ET_B_R and PHD2 expression are inversely correlates (Figure 3C). Moreover, to gain further insight into the mechanism through which ETs regulates PHD2 expression, we measured PHD2 mRNA in response to ET-1. As shown in Figure 3D, real-time PCR analysis indicated that ET-1 treatment inhibited PHD2 mRNA expression by ∼50% at the 6 and 8 h time points. To determine whether ETs-suppressed PHD2 mRNA expression is due to an effect on PHD2 transcription, we transfected melanoma cells with a luciferase gene reporter construct driven by the PHD2 promoter. ET-1 and ET-3 induced an inhibitory effect on PHD2 promoter, which after 8 h reached 45% of inhibition compared to the control, while BQ788 blocked this effect (Figure 3E and Figure S3A). To confirm the involvement of PHD2 on ETs-induced HIF-1α protein stability, we performed a reconstitution experiment by overexpressing each of the PHD-cDNA in 1007 cells. The overexpression of PHD1, PHD2 and PHD3 was confirmed by Western blotting (Figure S3B). HIF-1α and HIF-2α accumulation in response to ETs was specifically impaired in PHD2 overexpressing cells, indicating that re-expression of PHD2 is sufficient to counteract the ET-1- or ET-3-induced HIF-α expression (Figure 3F). These results identify the inhibition of PHD2 expression as the mechanism underlying ETs-induced HIF-α stabilization. Concomitantly to the block of HIF-α accumulation, the exogenous expression of PHD2 makes unable ET-1 and ET-3 to increase VEGF protein levels demonstrating a tight link between PHD2/HIF-α and ET-1-dependent VEGF expression (Figure 3F). Moreover, knockdown of PHD2 by inhibiting the prolyl hydroxylases with deferoxamine mesylate (DFO) resulted in a strong induction of HIF-α and VEGF expression. The addition of ET-1 to DFO did not induce a further increase in HIF-α, and VEGF protein, implying that ET-1 primarily regulates HIF-α protein accumulation through inhibition of PHD2 (Figure 3F). Furthermore, the luciferase activity of CMV-Luc-ODDD increased by ET-1 or ET-3 was impaired only in cells overexpressing PHD2 (Figure 3G), demonstrating that the re-expression of PHD2 antagonizes the effect of ET-1 and ET-3 on HIF-α degradation. These results further support the role of PHD2 on ETs-induced HIF-1α stability and angiogenic-related factor expression.

**Figure 3:** ETs decrease PHD2 expression and promoter activity. **A**. PHD1, PHD2 and PHD3 expression was analyzed in melanoma cells unstimulated (C) or stimulated with ET-1 for the indicated times. **B**. PHD2 protein expression was analyzed in cells stimulated as indicated for 24 h. **C**. Melanoma cells were treated with ET-1 and protein expression was analysed. **D**. 1007 cells were stimulated as indicated. Results are expressed as copy numbers of PHD2 transcripts over cyclophilin-A. Bars, ± SD. *, p<0.05 compared to the control. Inset shows PCR products for PHD2 and cyclophilin-A (CypA) **E**. Cells were transfected with the PHD2 promoter construct and stimulated as indicated for 8 h. Luciferase activity was expressed as fold induction. Bars, ± SD. *, p<0.006 compared to control; **, p<0.004 compared to ET-1. **F**. MOCK- and PHD1-, PHD2-, or PHD3-cDNA-transfected 1007 cells were stimulated with ET-1 or ET-3 for 16 h. Cells were treated with DFO alone or in combination with ET-1 and lysates were analysed for protein expression. **G**. 1007 cells were cotransfected with the CMV-Luc-ODDD construct and with the construct indicated in F, and stimulated with ET-1 or ET-3 for 16 h. Luciferase activity was expressed as fold induction. Bars, ± SD. *, p<0.001 compared to the control; **, p<0.005 compared to MOCK-transfected cells treated with ET-1 or ET-3.

### ETs signal through a PI3K-dependent ILK-AKT-mTOR pathway to induce HIF-1α stability and PHD2 inhibition

It has been reported that ILK, AKT and mTOR signalling are the main pathways controlling HIF-1α expression [6], [30], [31]. ILK is a serine/threonine kinase that plays an important role in linking extracellular signalling to the regulation of melanoma tumor growth and progression [30]–[33]. Therefore we analyzed the signalling pathways involved in ET-1-induced HIF-1α stability. In 1007 cells, ET-1 induced ILK protein expression (Figure 4A). Employing an immunocomplex kinase assay, we documented that ILK kinase activity was upregulated by ET-1 and inhibited by BQ788 demonstrating that ET_B_R is the relevant receptor in inducing ILK expression and activity (Figure 4A). Moreover, treatment with ET-1 induced phosphorylation of AKT and mTOR, and mTOR-downstream molecule p70S6k and p-4EBP1 (Figure 4A). These effects were blocked by BQ788 (Figure 4A), indicating that this effect occurs via ET_B_R binding. In 1007 cells treatment with the PI3K inhibitor, LY294002, or with mTOR inhibitor rapamycin, or transfection with a dominant negative ILK mutant (DN-ILK) suppressed the ET-1-induced HIF-1α, HIF-2α, and VEGF expression (Figure 4B), demonstrating that ET_B_R-induced HIF-1α and HIF-2α accumulation and VEGF expression in melanoma cells are mediated through a PI3K-dependent ILK/AKT/mTOR signalling. We further explored the decay of HIF-1α protein in melanoma cells treated with ET-1 in the presence of these signalling inhibitors. PI3K and mTOR inhibitors, as well as DN-ILK, inhibited the ET-1-mediated HIF-1α stabilization (Figure S4). LY294002, DN-ILK and rapamycin restored also the PHD2 promoter activity and PHD2 protein expression downregulated by ETs (Figure 4C,D). Altogether these results demonstrate that the inhibition of PHD2 progresses through an ET_B_R-mediated PI3K-dependent ILK/AKT/mTOR pathway to induce HIF-1α stability.

**Figure 4:** ETs-mediated PI3K–dependent ILK/AKT/mTOR pathway induces HIF-1α stability and PHD2 inhibition. **A**. Cell lysates from 1007 cells untreated (C), or treated with ET-1 alone or in combination with BQ788 were analyzed for ILK activity and for the indicated protein expression. ILK activity was indicated by the amount of 32P-labeling of MBP (pMBP). **B**. 1007 cells treated as indicated, were stimulated with ET-1 for 16 h and lysates were examined for indicated protein expression. **C**. PHD2 promoter activity was measured in cells transfected with the PHD2 promoter and treated as indicated for 8 h. Luciferase activity was expressed as fold induction. Bars, ± SD. *, p<0.001, compared to the control; **, p<0.005, compared to ET-1 or ET-3. **D**. PHD2 protein levels were analyzed in 1007 cells treated as indicated in B.

### PHD2 inhibition induced by ETs regulates angiogenesis and melanoma cell invasion

To determine whether the PHD2 inhibition induced by ETs was functionally involved in ET-1-induced effects regulated by HIF-α, we performed experiments targeting PHD2 in melanoma cells. siRNA against PHD2, similarly to ET-1 or ET-3, completely inhibited PHD2 protein with subsequent stabilization of HIF-1α and HIF-2α and increased VEGF levels that were not further increased by ETs (Figure 5A). To delineate the effect of PHD2 inhibition induced by ETs on angiogenesis, we measured the ability of endothelial cells to sprout forming three-dimensional structures resembling capillaries in response to conditioned medium from ET-1-treated cells silenced for PHD2. Conditioned medium from ET-1-treated 1007 cells promoted capillary branching of endothelial cells compared to untreated cells (Figure 5B). Interestingly, although knockdown of PHD2 enhanced tube formation, ET-1 treatment did not further enhance this angiogenic effect (Figure 5B). Next we determined whether secreted angiogenic factor regulated by PHD2 could explain the angiogenic effects induced by ETs. The secreted VEGF levels were increased by ET-1 or ET-3 as well as by PHD2 silencing, whereas no further increase was observed in ETs-treated PHD2-silenced 1007 cells (Figure 5C).

**Figure 5:** ETs regulate angiogenesis and melanoma cell invasion through inhibition of PHD2. **A**. Cell lysates from scRNA or siRNA for PHD2-transfected 1007 cells treated with or without ET-1 or ET-3 for 16 h were analyzed for protein expression. **B**. The ability of conditioned media from 1007 cells transfected and treated as in A, in inducing *in vitro* tube formation was analyzed on HUVEC. Results were represented as the number of cells in branch point capillaries. Bars, ± SD. *, p<0.001, compared to the scRNA control. **C**. Conditioned media from cells treated as in A were analyzed for VEGF secretion by ELISA. Bars, ± SD. *, p<0.001, compared to the scRNA control. **D**. 1007 cells were treated as in A and cell invasion was measured by chemoinvasion assay. Bars, ± SD. *, p<0.002, compared to the scRNA control.

Because invasive behaviour of melanoma cells is regulated by ETs through HIF-1α [25], we next examined whether PHD2 silencing could affect invasiveness. ETs or PHD2 siRNA promoted invasion in melanoma cells. ETs treatment of silenced PHD2 cells did not further increase cell invasion (Figure 5D), demonstrating that ETs signalling implies HIF-α-dependent angiogenesis and tumor cell invasion through PHD2 inhibition in normoxic conditions.

### ET_B_R blockade inhibits neoangiogenesis *in vivo*

In malignant melanoma microenvironment, ET_B_R has been shown to contribute to tumor progression by acting on both tumor and vascular endothelial cells [34], [35]. Indeed, ET-1 through ET_B_R promotes different steps of angiogenesis *in vitro* by acting directly on endothelial cells, as well as indirectly through VEGF [35], [36]. Immunostaining with anti-CD31, showed a significant (p = 0,0056) increase of the angiogenic response in the matrigels containing ET-1 (vessel numbers 20±1,4) compared to the control matrigels containing PBS (vessel numbers 1,5±0,3) (Figure 6A). In the plugs containing BQ788 and ET-1, the number of blood vessels was significantly (p = 0,0028) reduced (vessel numbers 1,5±0,2) compared to the matrigels containing ET-1 alone (Figure 6A). These results demonstrate that ET-1 selectively through ET_B_R promotes neoangiogenesis and that a selective ET_B_R antagonist can effectively impair angiogenesis *in vivo*.

**Figure 6:** ET_B_R blockade results *in vivo* in neovascularization inhibition, associated with reduced HIF-α and increased PHD2 expression. **A**. Matrigel sections containing PBS (C), ET-1, or BQ788+ET-1 were immunostained with anti-CD31 (arrows; original magnification ×160). **B**. Expression of indicated proteins was analyzed in M10 tumor xenografts by Western blot analysis. **C**. Tumors removed from control and A-192621-treated M10 xenografts were analyzed for PHD2 expression (original magnification ×250). **D**. Human metastatic melanoma tissues were analyzed for ET_B_R, PHD2, and HIF-1α expression (original magnification ×250).

### ET_B_R antagonist-induced decreased neovascularization is associated with reduced HIF-α and increased PHD2 expression in melanoma xenografts

We previously demonstrated that the treatment of nude mice bearing M10 xenograft with an orally active ET_B_R antagonist, A-192621, produces a significant (p<0,001) reduction of tumor growth [25]. Western blot analysis of tumors from M10 xenografts showed a significant reduction of HIF-1α, HIF-2α expression and an increase of PHD2 expression in A-192621-treated mice compared with the control, whereas no differences were observed in PHD1 and PHD3 expression (Figure 6B). Immunohistochemical evaluation of these tumors revealed a strong and homogenous increase in PHD2 expression levels (Figure 6C) compared to control, which paralleled the ability of A-192621 to reduce tumor vascularization, MMP-2 and VEGF expression [25]. These data underline the relevance of ET_B_R blockade in the regulation of tumor growth and neovascularization, resulting in down-regulation of VEGF and HIFα expression and increased levels of PHD2.

### Decreased PHD2 expression correlates with increased ET_B_R and HIF-1α expression in human melanomas

To further evaluate the relationship between PHD2, HIF-1α, and ET_B_R expression, we examined these protein in human primary (n = 6) and metastatic (n = 6) melanoma samples by immunohistochemistry. Of the twelve bioptic samples, eight had low PHD2 levels associated with high ET_B_R expression, thus indicating that the receptor and PHD2 expression are inversely correlated (p = 0.018). The expression of HIF-1α was very heterogeneous, most likely reflecting the fact that tumor microenvironment comprises areas of highly variable hypoxic and non-hypoxic regions. Figure 6D showed one of the 6 case of metastatic melanoma in which high ET_B_R expression, that occurs in clinically relevant situation [21], [22], was paralleled by high HIF-1α and low level of PHD2 expression. Taken together, our *in vivo* analysis suggest that ET_B_R expression significantly correlates with low PHD2 levels in melanomas, further supporting the potential clinical relevance that ET_B_R-mediated PHD2 downregulation may contribute to human melanoma tumorigenesis and progression through HIF-dependent pathways.

## Discussion

ET-1 axis represents one of the key regulators of tumorigenesis and tumor progression sharing with hypoxia the capacity to induce HIF-1α protein expression [25]–[28]. However, the mechanism underlying the regulation of HIF-1α mediated by ET-1 has been unexplored. In this study we demonstrate that in normoxia, ETs increase both HIF-1α and HIF-2α by preventing HIF-α protein proteosomal degradation through decreased PHD2 expression and that this regulation is critical to induce HIF-α-mediated VEGF expression, angiogenesis and tumor cell invasion. Blockade of ET_B_R, that inhibits tumor growth [25], results in an increased PHD2 expression concomitantly with a reduction of neovascularization and HIF-α expression *in vivo*.

Several growth factors, cytokines and hormones upregulate HIF-1α protein levels in normoxia by increasing HIF-1α gene transcription and/or mRNA translation without affecting protein stability [6]. Our results, concordantly with other studies [37], [38], demonstrate that non-hypoxic stimuli as ET-1, share mechanistic similarities with hypoxia regulating post-translational modifications (prolyl hydroxylation) resulting in increased HIF-1α stability. PHD2 is regarded as the main cellular oxygen sensor that regulates HIF-1α degradation in normoxia [10], [14], thereby suggesting that the inactivation of PHD2 may provide a critical mechanism in modulating HIF-1α. Until now very little information is available on the molecular control of PHD2. Our study reveals that ETs reduced PHD2 mRNA and protein expression and promoter activation, results in decreased HIF-1α hydroxylation. In melanoma cells treated with PHD2 inhibitor or in cells silenced for PHD2, ET-1 did not further increases HIF-1α or HIF-2α expression, angiogenesis and invasion, supporting that ET-1 regulates HIF-α-mediated effects through inhibition of PHD2. Moreover, the complete inhibition of ET-1-induced HIF-1α and HIF-2α accumulation observed in PHD2 overexpressing cells indicates that the re-expression of PHD2 is sufficient to counteract the effect of ETs. These results define the HIF-1α hydroxylase pathway as the link between ET-1 axis and the regulation of HIF-1α stabilization. Chan et al. [39] recently demonstrated that the loss of PHD2, observed in different tumor cells including melanoma, accelerates tumor growth and is associated with an induction of angiogenesis, suggesting that PHD2 is at the intersection of multiple complementary pathways regulating tumor growth. In this regard, our analysis of clinical melanoma samples, that express high levels of HIF-1α, reveals that ET_B_R activation is associated with a reduction of PHD2, further supporting that ET_B_R-mediated PHD2 downregulation represents a pathway for HIF-1α activation in human melanomas. Accumulating data have established that PHD2 is a direct HIF-1α target gene [40], [41]. Indeed PHD2 promoter contains HRE binding site responsible for the induction of human PHD2 gene by hypoxia [41]–[43]. It was therefore somewhat surprising to observe that ETs, which rapidly increased HIF-1α levels, inhibited PHD2 protein expression. This could be explained by recent results indicating that PHD2 induction generates an autoregulatory loop controlling HIF-1α stability [43]–[45]. Therefore our hypothesis supports the notion that ET-1 axis, similarly to hypoxia, modulates the autoregulatory loop of HIF-1α-PHD2 in melanoma cells through a balance between the inhibitory ET-1 and the stimulatory HIF-1α pathways for PHD2 transcription. In this context, we defined the intracellular signalling pathway that controls ET_B_R-induced PHD2 regulation in melanoma cells demonstrating that the inhibition of ILK/AKT/mTOR pathway antagonizes the ETs-induced HIF-1α stability and VEGF expression and restores PHD2 promoter activity and protein expression inhibited by ETs (Figure 7). As to whether this pathway is involved in controlling directly or indirectly PHD2, needs to be further characterized. The results demonstrating that knock-down of HIF-1α and HIF-2α makes both ETs and hypoxia unable to induce VEGF expression, implicate HIF as downstream check-point of interconnected signals induced by ET-1 axis and hypoxia, capable of modulating genes involved in tumor angiogenesis. Because the regulation of these factors is critical in the early stage of melanoma progression, one can envision that ET-1 axis, by mimicking hypoxia, can activate HIF-α enhancing the transcription of target genes, such as VEGF. As schematically described in Figure 7, ET-1 through ET_B_R-mediated signalling, stabilizes HIF-1α and enhances angiogenic factor expression, and hence angiogenesis, by inhibiting PHD2. Consistent with these results, it has been recently demonstrated that silencing of PHD2 induces neoangiogenesis *in vivo* by regulating the expression of multiple angiogenic factors through the stabilization of HIF-1α [46], [47]. In this regard, we demonstrated that *in vitro* tube formation of endothelial cells and melanoma cell invasion are regulated by ET_B_R in a PHD2-dependent manner. Taken together our findings disclose a yet unidentified regulatory mechanism, which relies on the role of ET-1 axis to promote tumor cell invasion, tumor growth and angiogenesis by decreasing PHD2.

**Figure 7:** A diagram of the signalling pathway activated by ET-1/ET_B_R axis in melanoma cells. Binding of ET-1 to ET_B_R leads to activation of PI3K–dependent ILK/AKT/mTOR signalling route, causing the inhibition of PHD2, thereby promoting HIF-1α stability, neovascularization and tumor cell invasion.

We recently identified HIF-1α/VEGF as downstream molecules of ET-1 axis in lymphangiogenesis [28]. In this scenario, it is possible to hypothesize that ET-1 through ET_B_R can stimulate angiogenesis and lymphangiogenesis via HIF-1α providing an alternative or complementary mechanism to the tumor hypoxic microenvironment. On support of this notion, in melanoma xenografts the reduction of tumor growth by ET_B_R blockade using the selective ET_B_R antagonist [25], was accompanied by reduction of tumor microvessel density, HIF-1α, HIF-2α and VEGF expression and a concomitant increase of PHD2 levels. In conclusion we demonstrated that ET-1 promotes melanoma progression by inducing HIF-α-mediated angiogenic signalling, through PHD2 inhibition. Thus ET_B_R antagonists, which have been shown to induce concomitant antitumor activity and suppression of neovascularization, may therefore represent a targeted therapeutic approach which is warrant to be explored in melanoma treatment.

## Materials and Methods

### Ethics Statement

The study was reviewed and approved by the ethical committee of Regina Elena National Cancer Institute. Written informed consent for tumor tissue archive collection and use in research was obtained from all melanoma patients prior to tissue acquisition under the auspices of the protocol for the acquisition of human tissues obtained from the Institutional Ethical Committee board (Official statement n.4 March 1^st^, 2006).

### Cells and cell culture conditions

The human cutaneous melanoma cell line 1007 was derived from primary melanoma [48]. The melanoma cell line SKMel28 (ATCC, Rockville, MD, HTB-72), M10, Mel120, and M14 [49] were derived from metastatic lesions. When the cells were exposed to hypoxia, oxygen deprivation was carried out in an incubator with 1%O_2_, 5%CO_2_, and 94% N_2_ and cells were growth for indicated times. Human endothelial cells were isolated from human umbilical vein endothelial (HUVEC), as previously described [34], and grown in complete Endothelial Growth Media. Melanoma cells were starved for 24 h in serum-free medium (SFM) then incubated for indicated times with either ET-1, ET-2 or ET-3 (100 nM; Peninsula Laboratories, Belmont, CA) or with unrelated scramble peptide B3 (IARVSTP) kindly provided by Dr. S. D'Atri [29] or with 100 µM deferoxamine mesylate (DFO; Sigma). The antagonists BQ788 (1 µM; Peninsula Laboratories, Abbott Park, IL) or A-192621 (1 µM; Abbott Laboratories) was added 15 min before agonists, whereas pre-treatment with MG132 (10 µM; Calbiochem, La Jolla, CA), cycloheximide (CHX, 20 µM; Calbiochem), LY294002 (25 µM; Cell Signalling, Beverly, MA), and rapamycin, (10 nM; Cell Signalling) was performed for 30 min before the addition of ETs. Serum-starved melanoma cells were transfected with 100 nM siRNA duplexes against PHD2 (Eurogenetec S.A Explera s.r.l AN, Italy), HIF-1α or HIF-2α or ET_B_R (ON-TARGETplus SMART pool, Dharmacon, Lafayette, CO) or with scrambled siRNA (scRNA) or positive control siRNA glyceraldehyde 3-phosphate dehydrogenase (GAPDH) obtained commercially (Dharmacon). Cell media were replaced with fresh SFM 48 h later and proteins were then extracted for HIF-1α, HIF-2α, and ET_B_R expression analysis. Conditioned cell medium containing secreted proteins was collected, centrifuged, filtered and concentrated.

### Western blot analysis

Whole cell lysates or homogenized M10 tumor specimens were subjected to SDS-PAGE and analyzed by Western blotting. Blots were developed with the enhanced chemiluminescence detection system (ECL; Amersham Pharmacia Biotech, Buckinghamshire, UK). Antibody against HIF-1α was from Transduction Laboratory (Lexington, KY). HIF-2α, PHD1, PHD2 and PHD3 antibodies were from Novus Biologicals (Littleton, CO), VEGF was from Santa Cruz Biotechnology (Santa Cruz, CA), ET_B_R was from Abcam plc (Cambridge, UK), GAPDH and β-actin, used as loading control, were from Oncogene (CN Biosciences, Inc., Darmastadt, Germany).

#### Real-time PCR

Total RNA was isolated using the Trizol (Invitrogen, Carlsbad, CA) according to the manufacturer's protocol. 5 µg of RNA was reversed transcribed using SuperScript® VILO™ cDNA synthesis kit (Invitrogen). Quantitative real-time-PCR was performed by using LightCycler rapid thermal cycler system (Roche Diagnostics, Indianapolis IN) according to the manufacturer's instructions. Reaction was performed in 20 µl volume with 0,3 µM primers, by using LightCycler-FastStart DNA Master Plus SYBR Green mix (Roche Diagnostics) from 1 µl cDNA. Primers used were as follow: PHD2, (forward) 5′-GCACGACACCGGGAAGTT-3′, (reverse) 5′-CCAGCTTCCCGTTACAGT-3′, Cyclophilin-A, (forward) 5′-TTCATCTGCACTGCCAAGAC -3′, (reverse) 5′–TGGAGTTGTCCACAGTCAGC-3′. The number of each gene-amplified product was normalized to the number of cyclophilin-A amplified product and expressed as copy numbers of PHD2 transcripts over cyclophilin-A (×10^−3^).

#### Transfectiona and luciferase assay

Transfection experiments employed the LipofectAMINE reagent (Invitrogen) according to the manufacturer's protocol. Plasmid for transfections were used as follow: 1 µg of ILK cDNA (kinase dead, DN-ILK) in pUSEamp (E359K mutant) (Millipore, Billerica, MA) or with pcDNA3-PHD1, pcDNA3-PHD2, or pcDNA3-PHD3 vectors (Dr. J. Geadle, The Henry Wellcome Trust Centre for Human Genetics, Oxford, UK) or empty vector pcDNA3 (MOCK) (Promega Corporation, Madison, WI) as control. 1007, and SKMel28 cells were transfected with different luciferase reporter constructs, including a plasmid encoding CMV-Luc- ODDD (Dr. R. K. Bruick, University of Texas Southwestern Medical Center, TX), or the previously described HRE-Luc construct (Dr. A. Giaccia, Stanford University School of Medicine, Stanford, CA), as well as the human PHD2 proximal promoter construct pGL3b (1454/3172) P2PWT (Dr. E. Metzen, University of Luebeck, Luebeck, Germany). The pCMV-β-galactosidase plasmid (Promega) was used as control for transfection efficiency. The cells were lysed and their luciferase activities were measured (Luciferase assay system, Promega).

#### ILK Immune Complex Kinase Assay

Integrin linked kinase (ILK) activity was measured as previously described [50]. Briefly cell lysates were immunoprecipitated with anti-ILK (Millipore). Assays were done directly on the protein A-Sepharose (Sigma) beads in the presence of 5 µCi of γ-^32^P (Amersham Pharmacia Biotech) and 2.5 µg of myelin basic protein (MBP) was used as substrate (Millipore). Phosphorylated MBP bands were visualized by autoradiography of dried SDS-10% PAGE gels.

#### ELISA

The VEGF protein levels in the conditioned medium were determined in triplicate by ELISA using the Quantikine Human VEGF immunoassay kit (R&D Systems, Minneapolis, MN).

#### *In vitro* Angiogenesis Assay

HUVEC were plated on basal membrane extract (10 mg/ml, Cultrex BME; Trevigen Inc. Helgerman, CT) in the presence of conditioned media from scRNA- or siPHD2-transfected 1007 cells. After 24 h, cells were visualized by light microscopy. The amount of angiogenesis was quantified by counting the number of cells in branch point capillaries (≥3 cells per branch) in five random fields per replicate.

#### Chemoinvasion assay

Chemoinvasion was assessed using a 48-well–modified Boyden's chamber (Neuro Probe Inc. Gaithersburg, MD) and 8 µm pore polyvinyl pyrrolidone–free polycarbonate Nucleopore filters (Costar, New York, NY) as previously described [25]. The filters were coated with an even layer of 0.5 mg/ml Matrigel (Becton Dickinson, Franklin Lakes, NJ). The lower compartment of chamber was filled with chemoattractant (ET-1 or ET-3). 1007 cells (1×10^6^ cells/ml) were harvested and placed in the upper compartment (55 µl per well). After 6 h of incubation at 37°C, the filters were removed, stained with Diff-Quick (Merz-Dade, Dudingen, Switzerland), and the migrated cells in 10 high-power fields were counted. Each experimental point was analyzed in triplicate.

#### M10 melanoma xenografts

Female athymic (*nu^+^/nu^+^*) mice, 4 to 6 weeks of age (Charles River Laboratories, Milan, Italy), were handled according to the Institutional guidelines under the control of the Italian Ministry of Health (DL 116/92), following detailed internal rules according to: Workamn P., et al. (1998) United Kingdom Coordinating Committee on Cancer Research (Guidelines for the welfare of animals in experimental neoplasia. Br. J. Cancer 77: 1–10). Mice were injected s.c. on one flank with 1.5×10^6^ viable M10 cells expressing ET_B_R. The mice were randomized in groups (*n* = 10) to receive treatment i.p. for 21 days with A-192621 (10 mg/kg/d), and controls were injected with 200 µl drug vehicle (0.25 N NaHCO_3_). The treatments were started 7 days after the xenografts, when the tumor was palpable [25]. Each experiment was repeated thrice, with a total of 20 mice for each experiment. All tumors for each group for each experiment were harvested from M10 xenografts for Western Blot analysis. Immunohistochemical analysis was performed in six samples of each group of the tumors previously analyzed by Western blot.

#### Matrigel plug assay

Male C57BL/6 mice (Charles River Laboratories) were handled according to the institutional guidelines under the control of the Italian Ministry of Health (DL 116/92), Mice were subcutaneously injected with 0.5 ml matrigel containing PBS (control), 0.8 µM ET-1 alone or in combination with 8µM BQ788, as previously described [34]. The matrigels surrounded by murine tissue were removed 10 days after implantation, and snap frozen in liquid nitrogen for immunohistochemical analysis.

### Immunohistochemistry

Indirect immunoperoxidase staining was carried out on acetone-fixed 4 µm tissue sections. The avidin biotin assays were performed using the Vectastatin Elite kit (for nonmurine primary antibodies) and the Vector MOM immunodetection kit (for murine primary antibodies) obtained from Vector Laboratories (Burlingame, CA) on size-matchable tumor tissues from control and A-192621 treated M10 xenografts [25] and on human melanoma samples. Sections incubated with isotype-matched immunoglobulins or normal immunoglobulins served as negative control.

### Statistical analysis

Results are representative of at least three independent experiments each performed in triplicate. Statistical analysis was done using the Student t test, Fisher's exact test, as appropriated. All analyses were performed using the SPSS 11 software (SPSS, Inc., Chicago, IL). All statistical tests were two-sided. p<0.05 was considered statistically significant.

## Supporting Information

Figure S1 ETs induce HIF-1α and HIF-2α expression in melanoma cells. A. 1007 cells were transfected for 48 h with scRNA or siRNA for ET_B_ R or siRNA for GAPDH, and ET_B_R or GAPDH protein expression was analyzed by Western blotting. B. Western blotting analysis of HIF-1α and HIF-2α expression was performed in whole cell lysates from 1007 and SKMel28 cells treated with increased concentrations of ET-1 for 16 h or with 100 nM ET-1 for the indicated times. C. Western blotting analysis of HIF-1α expression was performed in whole cell lysates from 1007 cells were treated with increased concentration ET-3 or with unrelated peptide scramble B3 (B3; 30 µM), for 16 h, or with 100 nM ET-3 for the indicated times. Anti-β-actin was used as loading control.
(0.24 MB TIF)

Figure S2 ET-1 impairs HIF-1α hydroxylation. 1007 and SKMel28 cells transfected with CMV-Luc-ODDD were treated with the indicated concentrations of ET-1 for 16 h. Luciferase activity was expressed as fold induction. Bars, ± SD. *, p<0.004, compared to control.
(0.05 MB TIF)

Figure S3 ET-3 decreases PHD2 promoter activity. A. 1007 and SKMel28 cells were transfected with the construct containing the PHD2 promoter and treated with 100 nM ET-3 alone or in combination with 1µM BQ788 for 8h. Luciferase activity was expressed as fold induction. Bars, ± SD. *, p<0.006 compared to control, **, p<0.005 compared to ET-1. B. 1007 cells were transfected with each of the pcDNA3-PHDs vectors or with pcDNA3 (empty vector, C). The expression of PHD isoforms was analyzed by Western blotting. Anti-β-actin was used as loading control.
(0.14 MB TIF)

Figure S4 ET-1-mediated PI3K-dependent ILK/AKT/mTOR pathway induces HIF-1α stability. 1007 or DN-ILK-transfected cells were stimulated with ET-1. Following 24 h, cells were stimulated with CHX for the indicated times with ET-1 alone or in combination with signalling inhibitors and analyzed for protein expression.
(0.12 MB TIF)
